RETRACTED

# The Effect of Renal Denervation on Cardiac Diastolic Function in Patients with Hypertension and Paroxysmal Atrial Fibrillation

**DOI:** 10.1155/2022/2268591

**Published:** 2022-05-28

**Authors:** Hai Xu, Zhixin Jiang, Wanying Jiang, Junyu Huo, Qijun Shan

**Affiliations:** ^1^Department of Cardiology, The First Affiliated Hospital of Nanjing Medical University, Nanjing, Jiangsu 222007, China; ^2^Department of Cardiovascular, The Affiliated Huaian No. 1 People's Hospital of Nanjing Medical University, Nanjing, Jiangsu 211103, China

## Abstract

**Objective:**

Renal artery denervation (RDN) can treat hypertension and paroxysmal atrial fibrillation (PAF). Hypertension and PAF can affect cardiac diastolic function. The study aimed to evaluate the effect of RDN on cardiac diastolic function in patients with refractory hypertension and PAF.

**Methods:**

190 consecutive patients with hypertension and PAF were recruited. The levels of NT-proBNP and metrics of echocardiography were measured before and after RDN in patients with refractory hypertension and PAF. The 190 patients were divided into the decreasing HR and nondecreasing HR group, the decreasing MAP and nondecreasing MAP group, the HFPEF group, and the normal diastolic function group, respectively.

**Results:**

Before RDN, the indices about cardiac diastolic function were out of the normal range. After RDN, the diastolic function improved in the indices of NT-proBNP, *E*/*e*′, *e*′. The diastolic function about the indices of NT-proBNP, *E*/*e*′, *e*′ was improved in the decreasing HR group, the decreasing mean arterial pressure (MAP) group, and the HFPEF group, correspondingly compared to the nondecreasing HR group, the non-decreasing MAP group, and the preoperative normal diastolic function group. In the multivariate analysis, the MAP and HR were the only two indicators significantly associated with the improvement of diastolic function.

**Conclusion:**

RDN could improve the diastolic function in patients with refractory hypertension and PAF. Patients with HFPEF could receive benefits through RDN. It was speculated that RDN improved the diastolic function mainly through decreasing HR and MAP.

## 1. Introduction

In the treatment of refractory hypertension, renal artery ablation (RDN) has become the most important nonpharmaceutical treatment modality [1–3]. By blocking the afferent and efferent nervous connections between the kidney and cerebra, the sympathetic nerve activity is inhibited and the hypotensive effect is achieved. With further study, RDN has been found to have significant therapeutic effects on other cardiovascular diseases, such as atrial fibrillation (AF), heart failure, and ventricular arrhythmia [4–9].

RETRACTED

Heart failure with preserved ejection fraction (HFpEF) was a common clinical disease, with an incidence rate as high as 50% in all heart failure cases [10–12]. Many factors are involved in the pathogenesis and progress of HFpEF. Hypertension and AF were the two common causes. Long-term hypertension, especially long-term uncontrolled hypertension, could directly lead to myocardial hypertrophy, myocardial wall stiffness, and compliance decline, eventually causing a decrease in diastolic function. AF could lead to the loss of atrial systolic function and ventricular irregular contraction and then promote the decline of cardiac diastolic function. Similar to persistent AF, paroxysmal atrial fibrillation (PAF) could also have a significant impact on cardiac diastolic function.

The patients with refractory hypertension and PAF simultaneously were common in clinical. RDN has a therapeutic effect on such patients. Theoretically, the RDN also has a certain effect on cardiac diastolic function in these patients. In this study, we studied the changes in diastolic function in patients with refractory hypertension and PAF before and after RDN.

## 2. Methods

### 2.1. Study Design

This was a single-center, prospective study. Patients were recruited for this study between January 2013 and December 2018 from the Department of Internal Medicine-Cardiovascular, the People's Hospital affiliated with Nanjing Medical University. Written informed consent was provided by all subjects before participation in study-related procedures. The study was approved by the Jiangsu Province People's Hospital Clinic Institutional Review Board, and the study was registered (NCT01418248). All patients were screened strictly before taking the study.

### 2.2. Process of RDN

Percutaneous femoral artery puncture with a modified Seldinger technique was performed under local anesthesia. Selective invasive left and right renal artery angiography was performed by using a JR4.0 catheter. Radiofrequency ablation was delivered using a cold brine temperature control ablation catheter through Z-shaped ablation from the left and right renal artery trunk to the proximal head. The ablation parameters were as follows: temperature (<45°C), impedance (<250 Ω), and power (10 W). The routine setting of the ablation energy was 10 W to start ablation. If the patient had difficulty tolerating pain in the process of ablation, the ablation energy would be reduced until the patient could tolerate it, and the target of energy and time were set as follows: 9.0–10 W for 60 s, 8.0∼9.0 W for 90 s, and < 8.0 W for 120 s. If the temperature exceeds 45°C or the impedance was over 250 Ω, the ablation was stopped and changed to the other suitable sites. The parameters of heart rate (HR) and MAP (1/3 systolic blood pressure + 2/3 diastolic blood pressure) were also recorded throughout the RDN.

RETRACTED

### 2.3. Definitions

#### 2.3.1. PAF

PAF is defined as atrial fibrillation (AF) episode recording by ECG or ambulatory electrocardiogram, lasting more than 5 minutes and less than 7 days, being reversed by medication or spontaneously. The secondary atrial fibrillation (due to cardiac surgery, infection, or hyperthyroidism) was excluded. In this study, heart rate was monitored mainly via ambulatory ECG. The Holter test was performed before RDN and during the follow-up period.

#### 2.3.2. Refractory Hypertension

The resistant hypertension was defined based on the 2018 American Heart Association Scientific Statement [13]. We defined resistant hypertension as clinic BP ≥140/90 mmHg using 3 antihypertensive medications, including a diuretic, or using ≥4 drugs regardless of having controlled or uncontrolled BP levels. The blood pressure was monitored mainly via ABPM. The ABPM was performed before RDN and during the follow-up period.

#### 2.3.3. HFpEF

The typical symptoms or signs of HF included fatigue, weakness, dyspnea, orthopnea, and edema. The diagnosis of HFpEF was established in patients with the above typical symptoms or signs, NT‐proBNP >450 pg/ml (<50 years), or >900 pg/ml (>50 years), the parameter of transthoracic echocardiogram (TTE), including left ventricular ejection fraction (LVEF) ≥50%, plus an *E*/*e*′ ≥13, and a mean *e*′ septal and lateral wall <9 cm/s [14–16].

### 2.4. Echocardiography

The parameters included LVEF, left ventricular end-diastolic diameter (LVEDd), and left atrial diameter (LA). Two-dimensional Doppler and tissue Doppler echocardiography were performed according to guidelines by experienced sonographers [15, 16]. Using the pulsed-wave Doppler technique, the peak flow velocity of the early rapid diastolic filling wave (E) and late diastolic filling wave (*A*) were measured. Using the tissue Doppler technique, early mitral annulus velocity (*e*′) was measured at the lateral and septal annulus.

The examination of echocardiography was performed before RDN and during the follow-up period. During the examination of echocardiography, the cardiac rhythm needed to be sinus rhythm. If the AF attacked, the examination would be delayed until the sinus rhythm was restored.

### 2.5. Follow-Up

All patients received follow-up six months and twelve months after RDN. Patients would be contacted by telephone or correspondence if the deadline of the follow-up exceeded more than seven working days. Patients were considered as loss to follow-up if the deadline exceeded more than 30 days.

RETRACTED

### 2.6. Statistical Analysis

All statistical tests were two-sided, and *p* < 0.05 was considered to be statistically significant. Numbers with percentages were used to summarize categorical variables. Mean and standard deviation was used to summarize the continuous variables, and the comparison between groups was performed by the *t*-test. Cox regression was used to determine risk factors for the change of diastolic function. All statistical analyses were carried out using Statistical Package for Social Sciences version 23.0 (SPSS Inc, Chicago, IL, USA) and GraphPad Prism version 6.

## 3. Results

### 3.1. Patients' Characteristics

A total of 190 consecutive patients were enrolled in this study. During the follow-up period, 14 patients were lost to follow-up. All the patients' characteristics, comorbidities, and oral medications are described in Table 1. All patients presented a higher heart rate (94.33 ± 5.63 bpm) and blood pressure (156.38 ± 11.36/99.55 ± 9.71 mmHg). Diuretics and beta-blockers were the top two in all antihypertensive drugs. New oral anticoagulants were more common than warfarin.

### 3.2. The Change of Diastolic Function before and after RDN

As shown in Table 2, during the 6th month and 12th month follow-up, mean arterial pressure (MAP) and heart rate decreased, and the diastolic function improved as demonstrated by the NT-proBNP, *E*/*e*′, and *e*′. The number of patients with heart failure symptoms decreased, but there was no significant difference compared to preoperation. During the follow-up, with decreasing HR and BP, all types of oral medications reduced, and only the calcium-channel blockers and diuretics were statistically significant compared to preoperation.

### 3.3. The Relationship between Diastolic Function and HR

According to the degree of HR decrease during the follow-up period, patients were divided into decreasing HR group and nondecreasing HR. The decreasing HR group referred to the decrease of HR ≥10 bpm during the follow-up compared to preoperation, while the nondecreasing HR group referred to the decrease of HR <10 bpm or the HR increasing. In order to eliminate the interference, those whose HR fluctuated in different groups during the two follow-up periods were excluded. The diastolic function in the decreasing HR group was improved during the 6th month and 12th month follow-up about the indices of NT-proBNP, *E*/*e*′, and *e*′. However, no significant change in parameters was observed about diastolic function in the nondecreasing HR group before and after RDN (Figure 1).

### 3.4. The Relationship between Diastolic Function and MAP

According to the degree of the MAP level during the follow-up period, patients were divided into the decreasing MAP group and the nondecreasing MAP group. The decreasing MAP group referred to the decrease of MAP ≥10 mmHg during follow-up compared to preoperation, while the nondecreasing MAP group referred to the decrease of MAP <10 mmHg or the MAP increasing. In order to eliminate the interference, those whose MAP fluctuated in different groups during the two follow-up periods were excluded. The diastolic function in the decreasing MAP group was improved during the 6th month and 12th month follow-up. Surprisingly, the improvement degree of heart function was less significant during the 6th month follow-up, and been significant during the 12^th^ month follow-up about the indices of NT-proBNP, *E*/*e*′, and *e*′. However, no significant change in parameters was observed about diastolic function in the nondecreasing MAP group before and after RDN (Figure 2).

RETRACTED

### 3.5. The Change of Diastolic Function and Basal Cardiac Function

According to the cardiac function before RDN, all the patients were divided into the HFPEF group (70 patients) and the normal diastolic function group (120 patients). Compared to preoperation, the diastolic function in the HFpEF group was improved about the NT-proBNP, *E*/*e*′, and *e*′ during the 6th month and 12th month follow-up. The relevant indicators showed no significant change the in normal diastolic function group before and after RDN (Figure 3).

### 3.6. Risk Factors for the Change of Diastolic Function

During follow-up, a total of 50 patients presented with an improvement of diastolic function. In the univariate Cox regression model, both MAP and HR were associated with the improvement of diastolic function. In the multivariate analysis, the MAP and HR remained to be significantly associated with the improvement of diastolic function (Table 3).

## 4. Discussion

The two main findings from this study are as follows: First, the cardiac diastolic function in patients with refractory hypertension and PAF could decrease. Second, RDN could improve the diastolic function in these patients.

Previous research found that 10% of hypertension could cause a cardiac diastolic function decline [17, 18]. Long-term hypertension, especially poorly controlled, could decrease the left ventricular compliance and increase stiffness [19–21]. AF could cause a variety of hemodynamic abnormalities such as rapid and irregular atrial activation impairing atrial contractile function, loss of regularity of atrioventricular conduction, and irregular ventricular contraction. These could further reduce the cardiac output and cause an increase in myocardial oxygen consumption, abnormal calcium regulation, myocardial remodeling, myocardial fibrosis, *etc* [22–24]. Thus, theoretically, the diastolic function in patients with refractory hypertension and atrial fibrillation could decrease. Some traditional indicators of cardiac diastolic function were not sensitive to distinguish the decline of heart function. But the latest indicators, such as NT-proBNP, *E*/*e*′, and *e*′, could help to improve the positive rate of HFPEF.

RETRACTED

The basic principle of RDN is to selectively destroy the renal sympathetic nerve fibers so as to decrease the peripheral norepinephrine secretion and play a hypotensive role. RDN inhibits the sympathetic nerve and RAAS activity, lowers the norepinephrine level, and decreases plasma AngII and aldosterone levels to play a role in the treatment of atrial fibrillation [25–28]. By lowering blood pressure and heart rate, RDN could improve left ventricular compliance, reduce left ventricular stiffness, and ameliorate atrial fibrosis and electrical remodeling by controlling blood pressure [29–32]. All these help to improve the cardiac diastolic function.

RDN had no effect on patients with normal diastolic function, but it could improve the diastolic function in those who had already suffered from a diastolic dysfunction decline. This phenomenon can be explained that the cardiac function of patients with hypertension and AF was still in the compensatory stage before RDN. Through RDN, the therapeutic effect of lowering blood pressure and heart rate was achieved. However, the effect of improving cardiac diastolic function could not be reflected, because diastolic function was within the normal range before RDN. Therefore, it was reasonable to speculate that the improvement of diastolic function of patients through RDN was mainly concentrated on those who had already suffered from diastolic dysfunction.

The cardiac diastolic function was improved in the decreasing HR group and the decreasing MAP group during the 6th month and 12th month follow-up. RDN could reduce both the HR and MAP simultaneously. As the heart rate is declining, the cardiac cycle and diastolic period prolonged, which could directly affect diastolic function. As MAP decreases, the left ventricular compliance and stiffness would improve. It was speculated that RDN improved the diastolic function mainly through decreasing the HR and MAP. In Cox regression analysis, only the MAP and HR remained to be significantly associated with the improvement of diastolic function.

This was a single-center study with a small sample size. We did not take a sham-operated group as a control, because of the sample size, short follow-up time and the condition were limited. Patients with different baseline complications might also be involved in diastolic dysfunction. The diastolic function was evaluated mainly by NT-proBNP and echocardiography, instead of a more accurate invasive examination method, such as CAP, PCWP, and CO. We took the change of 10 bpm and 10 mmHg as the clinically significant boundaries in HR and MAP. The first reason was that similar indicators were used to evaluate the effect of RDN in the past. The other reason was that the sample size of this study was too small to have further group discussion. The evaluation was based on the patients with refractory hypertension and atrial fibrillation, but we did not discuss separately. Oral medications have a certain impact on heart function, such as BB and ACEI/ARB, which were mainly used to control blood pressure and heart rate. However, after RDN, only diuretics and CCB had statistical significance in reduced oral medications. Regression analysis also showed that the factor of oral medications was not related to diastolic function.

RETRACTED

RDN could improve the diastolic function in patients with hypertension and PAF. The patients with HFPEF could receive benefits through RDN. It was speculated that RDN improved the diastolic function mainly through decreasing HR and MAP.

## Figures and Tables

**Figure 1:** The relationship of cardiac function and HR. (a) The different change of HR during baseline, 6th month, and 12th month follow-up between the decreasing HR and nondecreasing HR group. (b) The level of NT-proBNP of the two groups. (c) The level of *E*/*e*′ of the two groups. (d) The change of e′ between the two groups. Values are given in the form of mean ± SD. ^*∗∗∗*^*P* < 0.001 versus the baseline group.

**Figure 2:** The relationship of cardiac function and MAP. (a) The different change of MAP during baseline, 6th month, and 12th month follow-up between the decreasing MAP and non-decreasing MAP group. (b) The change of NT-proBNP of the two groups. (c) The change of *E*/*e*′ of the two groups. (d) The change of e′ between the two groups. Values are given in the form of mean ± SD. ^*∗∗∗*^*P* < 0.001 versus the baseline group.

**Figure 3:** Changes of NT-proBNP, E/e' levels and e' levels in HFREF and normal group at baseline, the 6th month, and the 12th month. (a) NT-proBNP levels. (b) *E*/*e*′ levels. (c) *e*′ levels. Values are given in the form of mean ± SD. ^*∗∗∗*^*P* < 0.001 versus the baseline group.

**Table 1:** Patient characteristics.

Detection indexes	Patients (*n* = 190)
Age, y	53.21 ± 7.38
Male, *n* (%)	104 (54.73)
Currently smoking, *n* (%)	9 (4.73)
BMI (kg/m^2^)	24.33 ± 2.57
SBP (mmHg)	156.38 ± 11.36
DBP (mmHg)	99.55 ± 9.71
HR (bpm)	94.33 ± 5.63
Comorbidities, *n* (%)	
Respiratory diseases	2 (1.05)
Diabetes	7 (3.68)
Cerebrovascular disease	5 (2.63)
Renal insufficiency	4 (2.11)
Dyslipidemia	5 (2.63)
Medications, *n* (%)	
ACEIs/ARBs	126 (66.32)
Beta-blockers	163 (85.79)
Calcium-channel blockers	133 (70.00)
Diuretics	190 (100.00)
Amiodarone	32 (16.84)
Propafenone	10 (5.26)
Warfarin	21 (11.05)
NOACs	145 (76.32)

BMI: body mass index. Respiratory diseases include chronic bronchitis, emphysema, chronic obstructive pulmonary disease, asthma, and moderate and severe pulmonary hypertension. Cerebrovascular disease is defined as a history of stroke, cerebral hemorrhage, carotid artery stent, or angioplasty. Renal insufficiency is defined as serum creatinine eGFR <60 mL/min/1.73 m^2^. Dyslipidemia is defined as previous dyslipidemia or a history of anti-lipid medication. ACEIs/ARBs: angiotensin-converting enzyme inhibitors/angiotensin-receptor blockers; NOACs: novel oral anticoagulants.

RETRACTED

**Table 2:** Assessment of the cardiac structure and function in patients before and after RDN.

Detection indexes	Patients		
	Baseline (*n* = 190)	6 months (*n* = 184)	12 months (*n* = 176)
SBP (mmHg)	156.38 ± 11.36	133.57 ± 8.56^*∗∗∗*^	135.24 ± 7.27^*∗∗∗*^
DBP (mmHg)	99.55 ± 9.71	86.71 ± 6.68^*∗∗*^	85.61 ± 5.16^*∗∗*^
MAP (mmHg)	118.50 ± 9.87	102.33 ± 7.67^*∗∗*^	102.15 ± 6.87^*∗∗*^
HR (bpm)	94.33 ± 5.63	78.84 ± 6.36^*∗∗∗*^	79.37 ± 7.15^*∗∗∗*^
NT-proBNP (pg/ml)	458.67 ± 10.33	216.64 ± 9.75^*∗∗∗*^	221.69 ± 11.49^*∗∗∗*^
*E*/*A*	1.06 ± 0.06	1.07 ± 0.08	1.03 ± 0.06
*E*/*e*′	17.23 ± 1.21	11.23 ± 1.03^*∗∗∗*^	10.17 ± 1.09^*∗∗∗*^
*e*′ (cm/s)	5.77 ± 0.64	8.43 ± 0.84^*∗∗∗*^	7.27 ± 0.76^*∗∗∗*^

Values are given in the form of mean ± SD. ^*∗∗*^*P* < 0.001; ^*∗∗∗*^*P* < 0.001 versus the baseline group.

**Table 3:** Risk factors of the improvement of diastolic function.

Variables	Univariate		Multivariate	
	HR	*P* value	HR	*P* value
MAP	0.31 (0.29–0.39)	0.033	0.062 (0.031∼0.088)	0.043
HR (bpm)	0.006 (0.002∼0.013)	0.007	0.008 (0.003–0.014)	0.037
EGFR	0.006 (0.002–0.014)	0.122	—	—
Medications	0.01 (0.009∼0.015)	0.625	—	—

eGFR: estimated glomerular filtration rate; HR: heart rate; MAP: mean blood pressure. Medications referred to the changes of drugs categories.

## Data Availability

The data used to support the findings of this study are available from the corresponding author upon request.
